# SNHG6 modulates oxidized low-density lipoprotein-induced endothelial cells injury through miR-135a-5p/ROCK in atherosclerosis

**DOI:** 10.1186/s13578-019-0371-2

**Published:** 2020-01-07

**Authors:** Haiyan Shan, Dawei Guo, Siyang Zhang, Huimeng Qi, Shen Liu, Yanmei Du, Yini He, Bofu Wang, Ming Xu, Xiaosong Yu

**Affiliations:** 1 Department of General Practice, The First Affiliated Hospital of China Medical University, No. 155 Nanjing North Street, Heping District, Shenyang, 110001 China; 2 Department of the Fourth General Surgery, The Fourth Affiliated Hospital of China Medical University, No. 4 Chongshan East Road, Huanggu District, 110032 Shenyang, China; 3 Department of the Science and Experiment Center, The China Medical University, No. 77 Puhe Road, Shenbei New Area, 110122 Shenyang, China

**Keywords:** Atherosclerosis, SNHG6, miR-135a-5p, ROCK, Endothelial injury

## Abstract

**Background:**

Plenty of long non-coding RNAs (lncRNAs) play vital roles in the progression of atherosclerosis. Small nucleolar RNA host gene 6 (SNHG6) is a well known lncRNA that is aberrantly high expressed in atherosclerosis patients. However, its function and basic mechanism in atherosclerosis events have not been well clarified.

**Methods:**

The expression patterns of SNHG6, miR-135a-5p, ROCK1 and ROCK2 in clinical samples and cells were detected by RT-qPCR assays. Cell Counting Kit-8 (CCK-8), flow cytometry assays, ELISA and reactive oxygen species (ROS) and malondialdehyde (MDA) detection, were performed to assess cell viability, apoptosis, inflammation and oxidative stress, respectively. Western blot analysis was carried out to examine the protein levels of Bax, Bcl-2, and SNHG6. Luciferase reporter and RIP assays were used to confirm the true interaction between SNHG6 and miR-135a-5p, or miR-135a-5p and ROCK.

**Results:**

The levels of SNHG6, ROCK1 and ROCK2 were notably increased and miR-135a-5p was decreased in atherosclerosis patients and oxidized low-density lipoprotein (ox-LDL)-treated HUVECs. Knockdown of SNHG6 alleviated ox-LDL-induced injury of HUVECs, while this effect was partly reversed by miR-135a-5p inhibitor. Moreover, overexpression of ROCKs aggravated miR-135a-5p-alleviated atherosclerosis cell injury. SNHG6 contributed to ROCK expression through sequestering miR-135a-5p as a molecular sponge.

**Conclusion:**

SNHG6 functions as a promoter in atherosclerosis events by targeting miR-135a-5p/ROCK axis in ox-LDL-stimulated HUVECs. This finding will help to develop a novel therapeutic strategy for atherosclerosis.

## Introduction

Atherosclerosis continues a common chronic inflammatory vascular disorder with increasing morbidity and mortality worldwide, which should be responsible for the occurrence of diverse clinical manifestations, such as stroke, myocardial infarction, peripheral arterial disease and coronary heart diseases [1, 2]. Endothelial dysfunction is considered to be the major trigger for atherosclerosis events. Arterial endothelial cells, which normally resist the adhesion of leukocytes, can release intercellular adhesion factors that capture leukocytes to their surfaces when suffering from adverse stimuli, such as hypertension, hyperlipidemia and inflammation stimulus [3, 4]. Endothelial dysfunction induced by endothelial cells (ECs) damage contributes to the accumulation of cholesterol-containing oxidative low-density lipoprotein (ox-LDL) in the artery wall [5]. In turn, excessive retention of ox-LDL can further induce ECs apoptosis by increasing oxidative stress and inflammatory responses, which eventually lead to the occurrence and development of atherosclerosis [6]. Thus, elucidation of the molecular mechanism on how ox-LDL induced ECs injury may be helpful for developing an effective approach for atherosclerosis treatment.

Long non-coding RNAs (lncRNAs) are a class of transcripts larger than 200 nucleotides (nt) without protein-coding potential. Recently, lncRNAs have attracted a large number of attentions due to their involvements in various pathological processes, including cancers, neurodegenerative disorders and cardiovascular diseases (CVD). Plenty of lncRNAs have been demonstrated to involve in atherosclerosis events by regulating the function of ECs, macrophages, and vascular smooth muscle cells (VSMCs). For instance, elevated lncRNA H19 expression causes proliferation induction and apoptosis inhibition in human umbilical vein endothelial cells (HUVECs) and VSMCs by upregulation of p38 and p65 [7]. Silencing of lnc00113 markedly suppresses VSMCs and HUVECs proliferation, survival, and migration by inactivation of PI3K/Akt/mTOR pathway [8]. LincRNA-p21 exerts an atheroprotective role in atherosclerosis by recovering the function of VSMCs and mouse mononuclear macrophage cells [9]. Knockdown of lncRNA XIST partially alleviates ox-LDL-elicited ECs injury via regulation of miR-320/NOD2 axis [10].

Small nucleolar RNA host gene 6 (SNHG6) has been uncovered to serve as a promoter in the progression of various human cancers, including hepatocellular carcinoma [11], glioma [12], gastric cancer [13], and osteosarcoma [14]. Moreover, SNHG6 promotes the formation of ventricular septal defect via serving as a molecular sponge of miR-101 and activating Wnt-β-catenin pathway [15]. A previous study also demonstrated that SNHG6 is substantially elevated in the plaque of atherosclerosis patients relative to healthy people, indicating the potentially diagnostic and therapeutic values of this lncRNA in atherosclerosis [16]. However, the biological function and precise mechanism of SNHG6 involved in atherosclerosis events remained elusive. In this study, we found that the expression level of SNHG6 was significantly upregulated in the serum of atherosclerosis patients and ox-LDL-induced HUVECs. Furthermore, SNHG6 remarkably facilitated the injury of ox-LDL-activated HUVECs through regulation of miR-135a-5p/ROCK network, indicating that SNHG6 might be a promising target for atherosclerosis treatment.

## Methods

### Clinical specimens

Peripheral venous blood samples from atherosclerosis patients (n = 32) who were diagnosed by clinical symptoms and coronary angiography, and healthy donors (n = 20) without atherosclerosis disease, inflammation, autoimmune diseases, or malignancies were collected from The First Affiliated Hospital of China Medical University between March 2017 and October 2018. The clinical parameters of atherosclerosis patients and healthy donors were shown in Table 1. The serum was separated from blood samples by low-speed centrifugation and then stored at − 80 °C for subsequent study. This study was carried out in accordance with the approval of the Research Ethics Committee of the First Affiliated Hospital of China Medical University and written informed consent was signed by each participant prior to this study.

**Table 1:** Clinical parameters of atherosclerosis patients

Parameters	Normal controls	Atherosclerosis patients
Number	20	32
Sex (female, %)	33	46
Age	63.21 ± 7.21	60.25 ± 8.04
Total cholesterol (mmol/l)	3.46 ± 0.88	5.61 ± 0.58*
LDL-C (mmol/l)	2.32 ± 0.43	2.58 ± 0.37
HDL-C (mmol/l)	1.67 ± 0.36	1.86 ± 0.40
TG (mmol/l)	1.45 ± 0.26	2.03 ± 0.35*
Creatinine(mg/dl)	1.02 ± 0.21	1.21 ± 0.12

Mean ± S.D.

* *P *< 0.05

### Cell culture and transfection

Human umbilical vein endothelial cells (HUVECs) and human embryonic kidney (HEK) 293T cells were purchased from American type culture collection (ATCC, Manassas, VA, USA) and grown in complete medium consisting of RPMI-1640 (Gibco, Grand Island, NY, USA), 10% Fetal Bovine Serum (FBS) (Gibco) and 1% penicillin/streptomycin (Thermo Fisher Scientific, Rockford, IL, USA) at 37 °C, 5% CO_2_. When cells grew to 70–80% confluence, various concentrations or designated concentration of ox-LDL (UnionBiol, Beijing, China) were added and incubated for another 24 h.

Small interfering RNA (siRNA) targeting SNHG6#1 (si-SNHG6#1) and SNHG6#2 (si-SNHG6#2), miR-135a-5p mimics, miR-135a-5p inhibitor, and relative negative controls were obtained from Thermo Fisher Scientific. Overexpression plasmids for SNHG6, ROCK1 and ROCK2 were constructed in GenePharma Co., Ltd (Shanghai, China) by inserting the full-length sequences of genes into pcDNA 3.1 empty vector. HUVECs were seeded into 6-well plates and transfected with 60 nM oligonucleotides or 0.5 µg plasmids using lipofectamine 2000 reagent (Invitrogen, Carlsbad, CA, USA) according to manufacturer’s procedure.

### Reverse-transcription qPCR (RT-qPCR)

SNHG6, miR-135a-5p, ROCK1 and ROCK2 levels in clinical samples and cells were measured by RT-qPCR. In brief, total RNAs extracted by Trizol reagent (Thermo Fisher Scientific) were reversely transcribed into cDNA using M-MLV reverse transcriptase (Invitrogen) with random primers or miR-135a-5p-specific RT primers. Then, SYBR Green Real-Time PCR Master Mix (Thermo Fisher Scientific) and qPCR primers were utilized to detect the expressions of SNHG6, miR-135a-5p, ROCK1 and ROCK2. The results were calculated by 2^−ΔΔCt^ method with GAPDH (SNHG6, ROCK1 and ROCK2) or U6 snRNA (miR-135-3p) as internal references.

### CCK-8 assay

Cell viability was analyzed using a Cell Counting Kit-8 (CCK-8) (Dojindo, Tokyo, Japan) in line with manufacturer’s instructions. Briefly, HUVECs were seeded into 96-well plate for 48 h and viable cells were examined by incubation with CCK-8 reagent for 2 h under a designated condition. Then, absorbance at 450 nm was measured using a microplate reader to assess cell viability.

### Caspase-3 activity and flow cytometry analyses

Caspase-3 activity assay kit (Beyotime, Beijing, China) was used to determine the activity of caspase-3. In short, cell lysates were incubated with assay buffer and caspase-3 substrate Ac-DEVD-pNA at 37 °C for 2 h, followed by the detection of absorbance at 405 nm using a spectrophotometer. Then, caspase-3 activity was assessed by drawing standard curve with different concentrations of standards as the abscissa and related OD values as the ordinate.

Cell apoptosis was tested by flow cytometry analysis using Annexin V-FITC/PI Apoptosis Detection Kit (Beyotime) following the manufacturer’s protocols. Briefly, cells digested with trypsin (without EDTA) were washed with PBS and re-suspended in 100 μl 1× Binding buffer, followed by the addition of 5 μl Annexin V-FITC and 10 μl propidium iodide (PI). After incubated for 15 min in the dark, cell apoptosis was detected by flow cytometry (BD Biosciences, Franklin Lakes, NJ, USA) and the data were analyzed with FlowJo software (Stanford University, San Francisco, California, USA).

### Western blot assay

Total protein in HUVECs was extracted by using RIPA buffer (Thermo Fisher Scientific). After protein quantification, equal amount of protein was subjected to SDS-PAGE gel electrophoresis, transferred to PVDF membrane (Millipore, Bedford, MA, USA), and incubated with primary antibody against Bcl-2 (ab185002, Abcam, Cambridge, UK), Bax (ab32503, Abcam), ROCK1 (ab45171, Abcam), ROCK2 (ab71598, Abcam), or GAPDH (ab181602, Abcam). After that, the membrane was further incubated with goat anti-rabbit IgG conjugated with horseradish peroxidase (HRP) (ab6721, Abcam). Specific protein signals were tested using Pierce™ ECL Western Blotting Substrate (Thermo Fisher Scientific) and quantified using Image J software.

### Measurement of inflammation-related factors and intracellular ROS and MDA

The concentrations of interleukin-6 (IL-6) and tumor necrosis factor-alpha (TNF-α) in culture supernatant were determined using ELISA Kits (R&D Systems, Minneapolis, MN, USA) according to the manufacturer’s procedures, followed by the detection of absorbance at 450 nm using a microplate reader. The production of reactive oxygen species (ROS) and malondialdehyde (MDA) were tested by ROS Assay Kit and Lipid Peroxidation MDA Assay Kit (Beyotime, Shanghai, China).

### Luciferase activity and RNA immunoprecipitation (RIP) assays

Partial sequences of SNHG6, ROCK1, and ROCK2 carrying putative miR-135a-5p binding sites or mutated sites were subjected to PCR amplification and cloned into psiCHECK-2 luciferase vector (Promega, Madison, WI, USA), named as SNHG6-WT, SNHG6-MUT, ROCK1-WT, ROCK1-MUT, ROCK2-WT, and ROCK2-MUT. MiR-135a-5p mimics or miR-NC mimics were transfected into HEK293T cells along with wild-type or mutant luciferase reporter. About 48 h thereafter, cells were harvested and luciferase activity in each group was measured using Dual-Luciferase Reporter Assay System (Promega).

RIP assay was performed to further explore the interaction between SNHG6 and miR-135a-5p, or miR-135a-5p and ROCK1 or ROCK2 using Magna RIP™ RNA-Binding Protein Immunoprecipitation Kit (Millipore) and anti-Argonaute2 (anti-Ago2) (ab32381, Abcam) or anti-IgG antibody (ab133470, Abcam) following the instructions of manufacturer. Briefly, cell lysates were co-incubated with A/G magnetic beads together with anti-Ago2 or anti-IgG antibody. Following the removal of protein using proteinase K, the enrichments of SNHG6, miR-135a-5p, ROCK1 or ROCK2 in immunoprecipitated complex were examined by RT-qPCR assay.

### Statistical analysis

All data were analyzed using SPSS 20.0 and results were expressed as mean ± standard deviation (SD) from three independent experiments. Difference between two or more groups were analyzed using Student’s *t*-test or one-way analysis of variance (ANOVA), *P* < 0.05 was considered as statistical significance.

## Results

### SNHG6 is upregulated in atherosclerosis patients and ox-LDL-induced HUVECs

Firstly, the expression patterns of SNHG6 in the serum of 32 atherosclerosis patients and 20 healthy donors were investigated by RT-qPCR assay. As a result, SNHG6 expression was significantly upregulated in the serum of atherosclerosis patients relative to healthy donors (Fig. 1a). Next, we further explored the effect of ox-LDL on endothelial cells injury, and results showed that introduction of ox-LDL dose-dependently decreased HUVECs viability compared to untreated group (Fig. 1b). Moreover, a dose-dependent and time-dependent increase of SNHG6 expression was also demonstrated in ox-LDL-treated HUVECs compared to relative controls (Fig. 1c, d).

**Fig. 1:** SNHG6 expression was elevated in the serum of atherosclerosis patients and ox-LDL-induced HUVECs. **a** SNHG6 expression in blood samples from atherosclerosis patients (n = 32) and healthy donors (n = 20) was examined by RT-qPCR. **b**, **c** HUVECs were treated with various concentrations of ox-LDL (0, 10, 25, 50 µg/ml) for 24 h, then cell viability was detected by CCK-8 assay (**b**), SNHG6 expression was detected by RT-qPCR assay. **d** HUVECs were treated with 25 µg/ml ox-LDL for 0, 24, 48 h, 72 h, and then SNHG6 expression was tested by RT-qPCR. ^*^P < 0.05 and ^**^P < 0.01

### SNHG6 knockdown alleviates ox-LDL-induced injury of HUVECs in atherosclerosis

To investigate the role of SNHG6 in atherosclerosis events, two specific siRNAs targeting SNHG6 were employed for the loss-of-function assay and the efficiency of knockdown was initially proved in HUVECs by RT-qPCR analysis (Fig. 2a). Next, we observed that ox-LDL treatment resulted in an elevated expression of SNHG6 in HUVECs, and this action was reversed by the introduction of si-SNHG6#1 or si-SNHG6#2 (Fig. 2b). Functionally, CCK-8 analysis indicated that the inhibitory effect of ox-LDL on cell viability was apparently abolished by si-SNHG6#1 or si-SNHG6#2 (Fig. 2c). Moreover, ox-LDL-stimulated caspase-3 activity and cell apoptosis were blocked following SNHG6 knockdown, as demonstrated by caspase-3 activity assay and flow cytometry assay (Fig. 2d, e). Additionally, the inhibitory effect of SNHG6 knockdown on cell apoptosis was also confirmed by the decreased Bax level and the increased Bcl-2 level (Fig. 2f). Inflammation and oxidative stress are considered as two main events involved in atherosclerosis development. Next, we further explored whether SNHG6 regulated atherosclerosis progression via influencing inflammatory response and oxidative stress. The results showed that ox-LDL stimulation triggered a marked increase of IL-6, TNF-α, ROS and MDA production, whereas SNHG6 depletion weakened ox-LDL-induced inflammation and oxidative stress in HUVECs (Fig. 2g–j). In addition, we also overexpressed SNHG6 in ox-LDL-induced HUVECs, and the results revealed that SNHG6 overexpression aggravated ox-LDL induced injury of HUVECs, which was contrary to SNHG6 knockdown (Additional file 1: Figure S1). These findings suggested that knockdown of SNHG6 greatly alleviated ox-LDL-induced atherosclerosis events through inhibiting inflammatory and oxidative stress.

**Fig. 2:** Knockdown of SNHG6 alleviated ox-LDL-induced injury of HUVECs. **a** The abundance of SNHG6 in HUVECs transfected with si-NC, si-SNHG6#1 or si-SNHG6#2 was examined by RT-qPCR. HUVECs were transfected with si-NC, si-SNHG6#1, or si-SNHG6#2 and then treated with or without 25 µg/ml ox-LDL for 24 h. **b** The expression of SNHG6 was detected by RT-qPCR assay. **c** Cell viability was determined by CCK-8 assay. **d** Caspase-3 activity was measured using commercially-available kit. **e** Cell apoptosis was assessed by flow cytometry. **f** The expression of apoptosis-related protein Bax and Bcl-2 was examined by western blot assay. **g**, **h** The release of inflammatory cytokines IL-6 and TNF-α were assessed by ELISA assay. **i**, **j** The production of oxidative status markers ROS and MDA were determined using commercially-available kits. *P < 0.05 and **P < 0.01; ^#^*P *< 0.05 and ^##^*P *< 0.01

### SNHG6 modulates miR-135a-5p expression by serving as a molecular sponge of miR-135a-5p in HUVECs

A previous study revealed the involvement of miR-135a in atherosclerosis development [17]. Thereby, we speculated that SNHG6 participates in the progression of atherosclerosis possibly via sponging miR-135a-5p. Firstly, we confirmed that the expression of miR-135a-5p was significantly declined in the serum of atherosclerosis patients compared with that in healthy donors (Fig. 3a), and miR-135a-5p showed a negative correlation with SNHG6 expression (Fig. 3b). Then, HUVECs were treated with different concentrations of ox-LDL (0, 10, 25, 50 µg/ml) for 24 h, and RT-qPCR results showed that miR-135a-5p expression level was gradually decreased (Fig. 3c). Bioinformatics analysis by Microcode suggested that miR-135a-5p shared the complementary binding sequences with SNHG6 (Fig. 3d). Luciferase reporter assay was performed to further explore the interaction between SNHG6 and miR-135a-5p, and the outcome indicated that miR-135a-5p mimics obviously decreased the luciferase activity of SNHG6-WT reporter compared to miR-NC mimics group, but no significant change was observed on the luciferase activity of SNHG6-MUT reporter (Fig. 3e). Subsequent RIP assay displayed that both SNHG6 and miR-135a-5p was highly enriched by anti-Ago2 when compared with IgG antibody, hinting the endogenous interaction between SNHG6 and miR-135a-5p (Fig. 3f). We then performed RT-qPCR assay to investigate the mutual regulation between SNHG6 and miR-135a-5p expression in HUVECs. Interestingly, upregulation of SNHG6 with plasmid vector led to a noticeable decrease of miR-135a-5p level, but lack of SNHG6 with siRNAs showed a positive effect on miR-135a-5p expression (Fig. 3g). Furthermore, miR-135a-5p mimics or inhibitors transfection, respectively decreased or increased SNHG6 level in HUVECs (Fig. 3h). In a word, SNHG6 negatively regulated miR-135a-5p expression through direct interaction in HUVECs.

**Fig. 3:** The targeted interaction between SNHG6 and miR-135a-5p by complementary binding. **a** miR-135a-5p expression in blood samples from atherosclerosis patients (n = 32) and healthy donors (n = 20) was examined by RT-qPCR. **b** The negative correlation between SNHG6 and miR-135a-5p expression in atherosclerosis patients. **c** HUVECs were treated with different concentrations of ox-LDL (0, 10, 25, 50 µg/ml) for 24 h, then miR-135a-5p expression was measured by RT-qPCR. **d** Predicted binding sites between SNHG6 and miR-135a-5p, as well as the mutant sites in SNHG6-MUT reporter. **e** HEK293T cells were co-transfected with miR-135a-5p mimic or miR-NC mimics together with GAS5-WT or GAS5-MT reporter, followed by the detection of luciferase activity in each group. **f** RIP assay was carried out to examine the enrichment levels of SNHG6 and miR-135a-5p in IgG or Ago2 immunoprecipitation complex. **g** HUVECs were transfected with SNHG6, si-SNHG6#1, si-SNHG6#2, or relative control, and then miR-135a-5p level was tested by RT-qPCR. **h** HUVECs were transfected with miR-135a-5p mimics, miR-135a-5p inhibitors, or relative control, and then SNHG6 level was measured by RT-qPCR. *P < 0.05 and **P < 0.01; ^##^*P *< 0.01

### SNHG6 exerts its role in atherosclerosis events partially by sponging miR-135a-5p

Here, we further investigated the mechanism underlying how SNHG6 regulated atherosclerosis development by transfection of si-SNHG6#1 or/and miR-135a-5p inhibitors into ox-LDL-activated HUVECs. As presented in Fig. 4a, introduction of miR-135a-5p inhibitors significantly suppressed miR-135a-5p expression, which was reversed by si-SNHG6#1 (Fig. 4a). Functionally, silencing of SNHG6 notably induced cell viability and inhibited cell apoptosis in ox-LDL-treated HUVECs, reflected by the decreased caspase-3 activity, apoptotic rate and Bax expression, as well as increased Bcl-2 expression; whereas inhibition of miR-135a-5p abolished these effects (Fig. 4b–e). Additionally, the inhibitory effects of SNHG6 knockdown on IL-6, TNF-α, ROS and MDA expression were also overturned by miR-135a-5p inhibitors (Fig. 4f–i). Taken together, these data indicated that SNHG6 acted as a major regulator in atherosclerosis via interacting with miR-135a-5p.

**Fig. 4:** SNHG6 regulated ox-LDL-induced injury of HUVECs via interacting with miR-135a-5p. ox-LDL-induced HUVECs were transfected with si-NC, si-SNHG6#1, si-SNHG6#1 + miR-NC inhibitors, si-SNHG6#1 + miR-135a-5p inhibitors for 48 h. **a** The enrichment of miR-135a-5p was examined by RT-qPCR. **b** Cell viability was determined by CCK-8 assay. **c** Caspase-3 activity was assessed by using commercially-available kit. **d** Cell apoptosis was detected by flow cytometry. **e** The protein expression of Bax and Bcl-2 was examined by western blot assay. **f**, **g** The release of IL-6 and TNF-α were measured by ELISA assay. **h**, **i** The production of ROS and MDA were detected using commercially-available kits. **P < 0.01; ^#^*P *< 0.05 and ^##^*P *< 0.01

### ROCK1 and ROCK2 are two authentic targets of miR-135a-5p

Plenty of literatures validates that miRNAs exert function by suppressing the expression of target mRNAs. To explore the regulatory mechanism of miR-135a-5p in SNHG6-mediated atherosclerosis progression, the Targetscan online software was employed to identify the potential targets of miR-135a-5p. Results showed that the 3′UTR of ROCK1 and ROCK2 had some binding sites within miR-135a-5p (Fig. 5a). Next, luciferase reporter assay was carried out to confirm the actual binding between miR-135a-5p and ROCK1 or ROCK2. As expected, miR-135a-5p mimics markedly inhibited the luciferase activity of wild type ROCK1 or ROCK2 reporter in HEK293T cells, but luciferase activity of mutant ROCK1 or ROCK2 reporter had no significant change following miR-135a-5p mimics or miR-NC mimic transfetcion (Fig. 5b, c). Furthermore, RIP assay were performed to figure out the potential targets of miR-135a-5p in RNA-induced silencing complex (RISC) and results displayed copious enrichments of ROCK1, ROCK2 and miR-135a-5p in Ago2 immunoprecipitation complex (Fig. 5d, e). Our findings subsequently confirmed that introduction of miR-135a-5p remarkably suppressed the expression of ROCK1 and ROCK2, while knockdown of miR-135a-5p obviously promoted the protein expression of ROCK1 and ROCK2 in HUVECs (Fig. 5f). To explore the possible involvement of ROCK1 and ROCK2 in atherosclerosis events, their expression levels in atherosclerosis samples and cells were measured by RT-qPCR. As results showed in Fig. 5g, h, j and k, ROCK1 and ROCK2 expression were markedly elevated in ox-LDL-activated HUVECs and the serum of atherosclerosis patients versus relative control. Moreover, the negative relationship between miR-135a-5p and ROCK1 or ROCK2 expression was also validated by correlation analysis (Fig. 5i, l). These data suggested that miR-135a-5p could bind to ROCK1 and ROCK2 to decrease their expression in HUVECs.

**Fig. 5:** ROCK1 and ROCK2 were identified as the targets of miR-135a-5p. **a** Potential sites targeted by miR-135a-5p in the 3′UTR of ROCK1 and ROCK2. **b**, **c** Wild-type or mutant ROCK1 or ROCK2 reporter were co-transfected into HEK293T cells with miR-135a-5p mimics or miR-NC mimics, followed by the detection of luciferase activity. **d**, **e** RIP assay was performed to examine the enrichment levels of ROCK1, ROCK2 and miR-135a-5p in IgG or Ago2 immunoprecipitation complex. **f** HUVECs were transfected with miR-135a-5p mimics, miR-135a-5p inhibitors, or relative control, and then ROCK1 and ROCK2 protein levels were detected by RT-qPCR. **g**, **h**, **j**, **k** The abundance of ROCK1 and ROCK2 in ox-LDL-induced HUVECs and the serum of atherosclerosis patients were determined by RT-qPCR. **i**, **l** The inverse correlation between miR-135a-5p and ROCK1 or ROCK2 expression in atherosclerosis samples. *P < 0.05 and **P < 0.01; ^##^*P *< 0.01

### Restoration of ROCK1 and ROCK2 aggravates miR-135a-5p-allevitated injury in ox-LDL-induced HUVECs

Subsequently, we further investigated the effects of ROCK1 and ROCK2 on miR-135a-5p-mediated atherosclerosis progression. ox-LDL-stimulated HUVECs were transfected with miR-NC mimics, miR-135a-5p mimics, miR-135a-5p mimics + vector, or miR-135a-5p mimics + ROCK1. About 48 h thereafter, RT-qPCR was carried out for ROCK1 and ROCK2 expression analyses, and results showed that transfection of ROCK1 and ROCK2 with plasmid vector notably abolished the inhibitory effects of miR-135a-5p on ROCK1 and ROCK2 expression (Fig. 6a, b). Following functional analysis highlighted that miR-135a-5p addition stimulated cell viability while suppressed apoptosis, which was demonstrated by the decreased caspase-3 activity, apoptotic rate and Bax expression, as well as elevated Bcl-2 expression. However, these effects were remarkably abrogated following ROCK1 or ROCK2 restoration (Fig. 6c–f). Then we further assessed the effects of miR-135a-5p, ROCK1 and ROCK2 on inflammatory response and oxidative stress. As shown in Fig. 6g–j, the production of IL-6, TNF-α, ROS and MDA was remarkably decreased in ox-LDL-treated HUVECs transfected with miR-135a-5p mimics, while re-expression of ROCK1 or ROCK2 overturned the inhibitory effect of miR-135a-5p on IL-6, TNF-α, ROS and MDA expression. These findings suggested that miR-135a-5p hindered atherosclerosis progression via directly targeting ROCK1 and ROCK2.

**Fig. 6:** miR-135a-5p modulated ox-LDL-induced injury of HUVECs via targeting ROCK1 and ROCK2. ox-LDL-induced HUVECs were transfected with miR-NC mimics, miR-135a-5p mimics, miR-135a-5p mimics + Vector, miR-135a-5p mimics + ROCK1, or miR-135a-5p mimics + ROCK2. **a**, **b** The expression of ROCK1 or ROCK2 was examined by RT-qPCR. **c** Cell viability was measured by CCK-8 assay. **d** Cell apoptosis was detected by flow cytometry. **e** The protein expression of Bax and Bcl-2 was tested by western blot assay. **f** Caspase-3 activity was evaluated by using commercially-available kit. **g**, **h** The secretion of IL-6 and TNF-α were detected by ELISA assay. **i**, **j** The production of ROS and MDA were examined using commercially-available kits. **P < 0.01; ^#^*P *< 0.05 and ^##^*P *< 0.01

### SNHG6 positively modulates ROCK1 and ROCK2 expression via sponging miR-135a-5p

In present study, we performed RT-qPCR assay to explore the effects of SNHG6 and miR-135a-5p on ROCK1 and ROCK2 expression. As presented in Fig. 1a, knockdown of SNHG6 caused a decreased level of ROCK1 and ROCK2 protein, whereas inhibition of miR-135a-5p abolished the inhibitory effect of si-SNHG6 on ROCK1 and ROCK2 expression in ox-LDL-induced HUVECs. Moreover, we further confirmed the positive correlation between SNHG6 and ROCK1 or ROCK2 expression in the serum of atherosclerosis patients (Fig. 7b, c). Collectively, our study indicated that SNHG6 aggravated ox-LDL-induced injury in HUVECs via targeting miR-135a-5p to upregulate ROCK expression (Additional file 2: Figure S2).

**Fig. 7:** SNHG6 positively modulates ROCK1 and ROCK2 expression via interacting with miR-135a-5p. **a** ox-LDL-induced HUVECs were transfected with si-NC, si-SNHG6#1, si-SNHG6#1 + miR-NC inhibitors, si-SNHG6#1 + miR-135a-5p inhibitors, followed by the detection of ROCK1 and ROCK2 protein levels. **b**, **c** The positive relationship between SNHG6 and ROCK1 or ROCK2 expression in atherosclerosis samples. **P < 0.01; ^##^*P *< 0.01

## Discussion

Atherosclerosis is a complex chronic disease troubling a large number of people worldwide. ox-LDL is considered to be a risk factor involved in the initiation and development of atherosclerosis by facilitating foam cells formation, ECs dysfunction, plaque formation, and inflammatory response. As reported by Geng, ox-LDL stimulates the inflammation of monocytes by activating NF-κB and facilitating monocyte chemoattractant protein-1 (MCP-1) and interleukin-8 (IL-8) production [18]. Moreover, ox-LDL contributes to HUVECs dysfunction and VSMCs calcification [10, 19]. Consistent with previous studies, we also certified that ox-LDL treatment elicited HUVECs injury by suppressing cell viability. Although the role of ox-LDL in atherosclerosis events has been expounded, the underlying mechanism is still poorly understood.

Recently, a plenty of lncRNAs have been certified to be abnormally expressed in atherosclerosis and implicate in ox-LDL-induced endothelial injury, such as MEG3 [20], MALAT1 [21], and RNCR3 [22]. In the present study, we first disclosed that the abundance of SNHG6 was markedly elevated in atherosclerosis samples and ox-LDL-induced HUVECs. Silencing of SNHG6 with siRNA protected HUVECs from ox-LDL-induced injury by recovering cell function and alleviating inflammatory reaction and oxidative stress. Emerging study indicates that lncRNA can function as a molecular sponge for miRNA to restrain the binding of miRNA and its target gene, eventually leading to the derepression of mRNA. Thereby, we aimed to investigate the mechanism of SNHG6 involved in atherosclerosis events by searching for specific miRNAs. By performing bioinformatics, luciferase reporter, and RIP assays, we confirmed the potential interaction between SNHG6 and miR-135a-5p by base pairing. MiR-135a has been recognized as a common tumor suppressor and shows obviously low expression in several types of human cancers. As reported by Tang et al., decreased miR-135a was correlated with the poor overall survival and progression-free survival durations of epithelial ovarian cancer (EOC) patients [23]. Zhou et al. stated that miR-135a impeded the development of non-small cell lung cancer (NSCLC) through modulation of IGF-1/PI3 K/Akt signaling pathway [24]. Hemmesi et al. proposed that enforced expression of miR-135a inhibited the differentiation of cancer stem cells to medulloblastoma via targeting Arhgef6 [25]. In addition, the protective role of miR-135a in macrophages and ECs has been also confirmed. For example, miR-135a protected HUVECs against mechanical stretch (MS)-induced cell apoptosis, oxidative stress, and inflammatory reaction by interacting with PHLPP2 and inducing the activation of PI3K/Akt pathway [26]. MiR-135a overexpression repressed macrophage-derived foam cell formation, oxidative stress and inflammatory events via downregulating toll-like receptor 4 (TLR4) in atherosclerosis [17]. Similarly, our study also indicated that inhibition of miR135a-5p aggravated si-SNHG6-alleviated HUVECs injury by inhibiting cell viability and facilitating apoptosis, inflammation, and oxidative stress, which was in line with the previous studies.

Given that miRNAs exert their functions mainly by repressing the expression of target genes, thereby we further explored the regulatory mechanism of miR-135a-5p in atherosclerosis via searching for its target mRNA. The results showed that ROCK1 and ROCK2 were two potential targets of miR-135a-5p, which expressions were negatively regulated by miR-135a-5p in HUVECs. Rho-associated protein kinases (ROCKs) belong to the family of serine/threonine kinases that composed of two isoforms ROCK1 and ROCK2. Reliable evidences have confirmed that ROCKs function as vital regulators in various cellular biological processes, including proliferation, motility, shape, metabolism, and death via acting on the cytoskeleton. In addition, the implication of ROCK in vascular damage and atherosclerosis events has been also demonstrated. For instance, Rho and its effector ROCK participated in the pathophysiology of hypertension by enhancing the sensitivity of vascular smooth muscle to calcium [27]. FSD-C10 induced the increase of cell viability in ox-LDL-treated brain microvascular endothelial cells (BMECs) by reducing ROCK/MAPKs-mediated apoptosis [28]. ROCK activity was suppressed by high dose atorvastatin independent of cholesterol reduction in atherosclerosis patients, indicating the potential therapeutic value of ROCK in patients with atherosclerosis [29]. Inactivation of the Rho/ROCK pathway by statins recovered the endothelial function and attenuated vascular inflammation and atherosclerosis [30]. In our study, we demonstrated that exogenous addition of ROCK1 or ROCK2 aggravated HUVECs injury, which was alleviated by miR-135a-5p overexpression, indicating that ROCKs were beneficial to the progression of atherosclerosis. Furthermore, we observed that knockdown of SNHG6 reversed the inhibitory effect of miR-135a-5p inhibitors on ROCK expression in ox-LDL-treated HUVECs.

Though the role and the regulatory mechanism of SNHG6 in ox-LDL-treated HUVECs have been elucidated, there are some limitations in our study. The precise function of SNHG6 in atherosclerosis need be verified by a further in vivo experiment. In addition, we explored the effects on ox-LDL-treated HUVECs in a short term, while atherosclerosis is a chronic disease; the long-term effects of SNHG6 on ox-LDL-treated HUVECs also need further study.

## Conclusion

In summary, our study firstly confirms that SNHG6 depletion protects HUVECs from ox-LDL-induced injury via regulation of miR-135a-5p/ROCK pathway. These findings raise the possibility that SNHG6 may be used as a potential therapeutic target for atherosclerosis prevention.

## Supplementary information

**Additional file 1: Figure S1.** Overexpression of SNHG6 aggravates ox-LDL-induced injury of HUVECs. (A) The abundance of SNHG6 in HUVECs transfected with Vector or SNHG6 was examined by RT-qPCR. HUVECs were transfected treated with or without 25 µg/ml ox-LDL for 24 h or transfected with vector or SNHG6 under ox-LDL treatment. (B) The expression of SNHG6 was detected by RT-qPCR assay. (C) Cell viability was determined by CCK-8 assay. (D) Cell apoptosis was assessed by flow cytometry. (E) The expression of Bax and Bcl-2 was examined by western blot assay. (F and G) The release of inflammatory cytokines IL-6 and TNF-α were assessed by ELISA assay. (H and I) The production of oxidative status markers ROS and MDA were determined using commercially-available kits. *P < 0.05 and **P < 0.01.

**Additional file 2: Figure S2.** SNHG6 aggravates ox-LDL-induced injury of HUVECs through targeting miR-135a-5p to regulate ROCK1 and ROCK2 expression.

## Data Availability

All data and materials about this work are available.

## Abbreviations

ECs: endothelial cells
CVD: cardiovascular diseases
VSMCs: vascular smooth muscle cells
HUVECs: human umbilical vein endothelial cells
FBS: Fetal Bovine Serum
RT-qPCR: reverse-transcription qPCR
RIP: RNA immunoprecipitation
